The article "Medical Health Data-Driven Physical Education Scheme: Public Environment-Oriented Exercise Health Management" was published in 2022. Journal: J Environ Public Health.

# Medical Health Data-Driven Physical Education Scheme: Public Environment-Oriented Exercise Health Management

**DOI:** 10.1155/2022/6399603

**Published:** 2022-07-31

**Authors:** Nan Yue

**Affiliations:** College of Physical Education, Beihua University, Jilin 132013, China

## Abstract

Smart wearable devices can encourage users to take an active part in exercise to a certain extent. The most important reason is that their entertainment function can bring users a better exercise experience, which is also one of the reasons why most people wear smart wearable devices during exercise. Another reason is that the medical and health data feedback of smart wearable devices can play a stimulating role, which is also the motivation of this study. Through the feedback of health data, students can perceive their own exercise situation, and teachers can plan more targeted exercise courses based on medical and health data, so as to improve the quality of physical education. This paper studies the origin and development of health data-driven learning; clarifies the logical mechanism between health data-driven learning and physical education; analyzes the internal needs of physical education design; discusses the characteristics of thinking, process, tools, and other elements of health data-driven learning in the new era of physical education reform; and carries out physical education teaching practice. Experiments have proved that health data-driven physical education is beneficial for improving students' emotional attitude and values, optimizing learning process and methods, and strengthening knowledge literacy and exercise skills. However, in today's poor public environment, the medical and health data-driven physical education scheme proposed in this paper is also applicable to the public-oriented exercise health management. Medical Health; Public Environment; Health Management; Data Analysis.

## 1. Introduction

The physical health level of students is directly related to the development of society, the future of the country, and the future of the nation. However, in recent years, the national student physical health monitoring shows that the physical health of Chinese students has been declining yearly, mainly manifested as a low vital capacity index, obesity, myopia, and poor stamina [1–3]. There are many ideas to solve students' physical health problems, but the key point is to start with physical education. This is because the main exercise time and space of students are in the school, while improving students' health is also the primary goal of physical education.

As an important component of school teaching system and the central position of school sports work, physical education has many functions such as guiding students to form good habits, exercising strong physique, developing sports skills, and shaping strong character [4, 5]. Under the background of modernization of education and acceleration of digitalization of sports in the new era, systematic promotion of physical education teaching reform in schools bears an important historical mission and social responsibility [6–8]. To improve the intelligence level of physical education teaching, it is necessary to further strengthen the sports teaching reform and innovation, make full use of and integrate the modern information technology, analyze and use data efficiently, actively promote the application practice of data-driven learning in physical education in schools, and promote the two-way integration of physical learning and physical education to achieve new results. In the era of rapid development of science and technology, distance teaching and multimedia teaching have been widely used in the teaching of various subjects and have achieved remarkable results. Therefore, we can also apply them to physical education teaching. Intelligent distance multimedia physical education not only provides great help for teachers and students, but also stimulates students' interest in learning physical education.

As wearable device technology is getting to be more mature, all kinds of wearable device products will enter the commons' daily life. At the same time, the rapid expansion of smart medical care and mobile medical care makes the application prospect of wearable devices in the medical and health field broader [9–11]. It is the increasingly extensive application of wearable devices in the field of medical and health that makes the health data-driven physical education scheme possible. Health data-driven is an inevitable choice for the development and reform of physical education in the new era [12, 13]. First, with the constant emergence of newly developing information technologies such as social media and iteration, the new era of digital development has brought new opportunities for the teaching reform of physical education innovation, making health data-driven learning and integration development a new trend of physical education. The innovation of student-oriented and student-friendly teaching mode driven by health data not only strongly supports the concept of student-centered education, but also fully exerts the significant advantages of health data-driven learning in reducing teaching costs, improving learning efficiency, and consolidating learning quality. Afterwards, health data-driven learning is a favorable way for the development of physical education. By effectively recording and feeding back the health data of the development of students' sports ability, students can participate more in sports learning and have a stronger sense of experience, which is conducive to the formation of deeper knowledge understanding and cultivation of reflective learning ability and promotes the qualitative change of sports learning. Finally, health data-driven learning is an innovative step in the development of physical education. A large number of practices have proved that health data-driven learning consolidates and strengthens physical education teaching through online and offline learning; effectively guarantees learning opportunities and learning fairness; and develops diversified teaching organizations, personalized teaching evaluation, three-dimensional teaching content, and other ways to reflect the multidimensional goals of education.

As the inheritance and sublimation of digital learning and mobile learning, health data-driven learning emphasizes the use of technology as a cognitive tool rather than a teaching tool to make learning more flexible and inclusive. With the extension of teaching paradigm from experience imitation to data-driven teaching, the systematic connection of curriculum system, the teacher-student interaction and integration, the evaluation and supervision of academic quality, and the reasonable creation of teaching situation in physical education need the help of health data-driven technology. However, with the development of China's economy and society and the advancement of urbanization, citizens pay more and more attention to the quality of life, and urban public environmental health has begun to attract public attention. Whether the health data-driven physical education scheme is suitable for public environment-oriented exercise health management will also be studied in this paper.

The remainder of the paper is structured as follows. Health data-driven-oriented innovation in physical education is studied in Section 2. In Section 3, practice and effect of health data-driven physical education are discussed. In Section 4, the development of health data-driven physical education is studied. Finally, the conclusion of this paper is given.

## 2. Health Data-Driven-Oriented Innovation in Physical Education

### 2.1. Health Data-Driven Thinking-Guided Innovation of Physical Education

Health data-driven physical education is not to reconstruct the teaching mode but is a process of integrating and optimizing sports skill teaching with technical tools. According to the theoretical framework of data-driven learning, the health data-driven physical education teaching model takes the teacher-student community as the main body, closely revolves around the basic structure of physical education classroom teaching, and fully exerts the four functions of data (Figure 1), in which the teacher-student community is the dual subject composed of teachers and students and resources, teaching, and experience construct the whole process of optimization and improvement of physical education teaching cycle in school during data-driven process.

The teacher-student community is not only the direct stakeholder of physical education teaching under data-driven learning, but also the executor of the teaching model [14, 15]. Under this framework, teachers make preparations based on the health data acquired by wearable devices. In other words, teachers are the subjects of health data collection and health data analysis. Students finally realize sports behavior change based on experience and are the object of health data decision-making and feedback. This model can promote the meaningful dialogue between teachers and students and the concerted action based on common goals, and it can accelerate the construction of democratic, equal, interactive, harmonious, and dynamic teaching atmosphere. Through health data-driven physical education, students can self-regulate their learning activities and acquire all kinds of learning resources on demand, which can promote the reconstruction and definition of the community of teachers and students in school physical education curriculum and enhance the relationship between teachers and students to return to the intrinsic nature.

### 2.2. Health Data-Driven Process-Guided Innovation of Physical Education Strategy

Health data acquisition, health data analysis, health data decision-making, and health data feedback constitute the power chain of health data-driven physical education. Health data acquisition is the foundation, health data analysis and health data decision-making are the key, and health data feedback is value presentation.

Medical health wearable devices refer to portable electronic devices which are used in daily life, exercise, health maintenance, and clinical medical activities and can be directly worn on the body or implanted into the human body [16–18]. They can sense, record, analyze, regulate, intervene, and even treat diseases and maintain health status through software support and data interaction. Medical health wearable devices are applicable to a wide range of people, with various types and complete functions. They not only have the functions of step counting, tracking daily activities and dietary habits, monitoring vital signs, and drawing electrocardiograms in real time, but also can monitor the health status of patients in real time and multiple dimensions. Health data acquisition refers to the process where wearable devices users collect personal identification data (height, weight, gender, date of birth, etc.), physiological data (blood sugar, blood pressure, heart rate, body temperature, etc.), and surrounding environment data (noise, temperature, humidity, pollution index, location, etc.) through sensors and circuit chips during medical health activities [19, 20].

The health data-driven dynamic chain is helpful in the overall consideration of the order of teaching contents, the procedure of teaching activities, the form of teaching organization, the use of teaching methods, and the utilization of teaching resources by strengthening the existing structure of physical education teaching activities. By obtaining more information of physical education status, it is beneficial to distinguish the subjective and objective conditions and status of teaching, especially the individual differences, and then realize the order and operability of teaching. At the same time, compared with the closeness of traditional physical education teaching, health data-driven learning pays more attention to the openness of physical education [21]. Through visual and data-based sharing of teaching information, it promotes communication and cooperation between subjects and objects, strengthens the deep body experience, highlights the individual characteristics of self-body perception, promotes the subjectivity in the learning process, and better exerts the initiative of learning [22, 23]. Health data-driven learning ensures the process management of teachers' teaching supervision in physical education and makes teachers' guidance play a better role, so as to realize the purpose of teaching students according to their abilities and innovation of physical education strategies.

### 2.3. Health Data-Driven Tools-Guided Innovation of Physical Education Methods

Health data-driven physical teaching has the advantages of planning process, adjusting rhythm, and expanding space. In the preparation part of physical education, it is helpful to optimize and promote the students' self-study behavior by sorting out the knowledge content carefully, decomposing the knowledge content, and realizing the individualized setting of learning objectives [24]. It is also helpful to make rational decisions to realize the learning task goal by dividing the learning points, helping the students to do a good job in exercise learning, and gradually crossing the stage platform period of exercise ability development, thus cultivating the lifelong exercise awareness [25]. At the same time, stereoscopic content recognition is conducive to opening the teaching boundary of physical education and promoting the integration of internal and external classroom. In the basic part of teaching, through real-time monitoring and acquisition, analysis of physical and mental state, and targeted guidance of teaching supervision, it is helpful to strengthen quality control and adjustment of students' physical education learning process, to achieve rational planning of learning task exercise through scientific training guidance and supervision, to help students strengthen physical exercise action and to consolidate their mastery of new knowledge and skills. Diversified teaching interaction also helps and supports flexible sports teaching and provides a multi-integrated form of full participation in learning. After physical education teaching, the learning effect will be accurately assessed by timely monitoring, analysis, and evaluation of learning quality and progress. In this way, it can assist students in developing reflective thinking and self-awareness [26]. It is necessary to make up for the limitations and shortcomings of body experience and realize the standardization and unification of teaching methods and learning methods, so as to generate positive interaction between body cognition, alternation of learning and practice, and skill formation, thus realizing the innovation of physical education teaching methods with the help of information technology.

## 3. Practice and Effect of Health Data-Driven Physical Education

### 3.1. Practice

For health data-driven physical education, emotional attitude and values are the internal motivation of learning, process and method are important links of learning, and knowledge and skills are the specific embodiment of learning ability and learning results. The study was divided into three groups: experimental group 1 (E1), experimental group 2 (E2), and control group (C1). Among them, E1 and E2 were health data-driven physical education courses conducted with wearable devices, with 20 subjects in each group. The difference between them is that the subjects of E1 is students, while E2 is exercise health management for public environment; that is, 20 citizens are randomly selected for participation. In C1, 20 subjects were randomly selected for traditional physical education without health data. Without affecting the teaching order, the whole experiment lasts 8 weeks and takes long jump once a week to compare the actual effect of health data-driven physical education with traditional teaching so as to prove the feasibility and effectiveness of health data-driven learning in physical education.

In the data acquisition process, electrocardiography (ECG) of E1 and E2 was collected. It is a time-based recording of the electrophysiological activity of the heart through the thorax to help diagnose arrhythmias, myocardial ischemia, myocardial infarction, etc. and to improve the safety of physical education. Pulse, blood pressure, blood oxygen, skin temperature, and body temperature of E1 and E2 were also collected. In addition, physical education mainly detects exercise, including automatic recognition, tracking, and energy consumption. Through real-time analysis of data collected by E1 and E2, the subjects were given targeted physical education. In the data decision-making process, retrospective comparison method [27] was used. Data feedback uses teaching feedback card and development record table. Each of E1 and E2 subjects receives the last class teaching feedback card before class, including key action screenshots, key action data, medical health data, teachers' evaluation and suggestions, and students' self-evaluation and thinking. Data for eight consecutive weeks are finally summarized and fed with technical action development record table, which is finally evaluated by the teachers. The control group was taught in traditional mode without data analysis and feedback. Teaching and evaluation are carried out by teachers with senior titles and more than 10 years of teaching experience. Before and after the experiment, three groups are surveyed with questionnaires on learning evaluation status and evaluated with long jump results. The learning progress and learning content of E1, E2, and C1 are synchronized, and their specific performance is shown in Table 1.

### 3.2. Practice Results and Analysis

#### 3.2.1. Health Data-Driven Physical Education Helps Promote Students' Emotional Attitudes and Values

As the result data of the long jump is fed back to the students regularly, combined with their own graphics and movement evaluation and analysis, it not only triggers the students' self-thinking, but also provides a basis for the adjustment of the practice goal in the next class, which effectively mobilizes the students' learning enthusiasm, strengthens their motivation, and stimulates their motivation. Stimulated by successful experience, slight but definite progress increases students' confidence, interest in learning, and desire for knowledge and actively exerts willpower to overcome side effects such as uncomfortable actions and unclear points caused by adjustment, so as to improve the effectiveness of the classroom and improve students' willpower quality simultaneously. Additionally, by analyzing the collected health data, teachers may determine whether students' exercises are standardized or tolerated by their bodies, allowing them to guide students to finish movements more scientifically and develop targeted physical education courses for students.

Although there are no significant differences in other indexes, the correlation indexes have mutual effects; for example, E1 and E2 are higher than C1 in the indexes of “physical ability,” “number of participation activities,” and “confidence level.” The overall results of E1 and E2 in the final assessment are better than those of the control group. Under the collaboration of common data, students acquire more obvious experience through health data-driven learning. Small changes of individuals gradually shape the overall environment in the process of gradual unification. The formation of a good learning atmosphere is also more conducive to the consistent growth of ability. Students enjoy gaining good experience in the process. The research shows that health data-driven physical education is more conducive to the development of students' attitude awareness and improvement of self-efficiency under the progressive processing of information.

#### 3.2.2. Health Data-Driven Physical Education Helps Optimize Students' Learning Process and Methods

By observing the process records, it was found that “shared language” and “shared movement” gradually appeared in the middle and later stages of the experiment. The appearance of “shared language” indicates that students' emotions have changed and resonated with each other, which is externally expressed as the desire to improve their scores, leading to the appearance of “shared movement.” “Shared language” and “shared movement” jointly lead to a change in students' exercise behavior. The students' recognition of movement is not only reflected in their own movement, but also in their concern for others' movements. Specifically, E1 is significantly higher than E2 and C1 in the frequency of observing and imitating others' long jump behavior. Especially in E1, a small discussion group of 2-3 students will be formed to compare and correct each other's technical actions. It can be seen that the health data-driven physical education affects students' way of thinking and communication and improves students' sense of identity to physical education through the sharing of common data.

Compared with traditional teaching, health data-driven physical education teaching creates a free physical education learning space for students, improves the way of students' physical education learning, and makes physical education classroom teaching more dynamic. Students are endowed with more autonomy in class. While accepting the “charm” of data, students are driven by health data, which further stimulates the freshness of students' exploration and their strong desire to keep trying [28]. Health data-driven physical education makes the use of teaching methods and means gentler for physical education teachers. Teachers can guide and control the classroom more freely and have more time to teach according to their aptitudes. As a result, classroom efficiency has been significantly improved. The role of teachers in the classroom has really become a cooperative role because of technological innovation [29, 30]. Teaching relationship is more democratic, more equal, and closer to the development trend of modern education.

#### 3.2.3. Health Data-Driven Physical Education Helps Enhance Students' Knowledge and Exercise Skills

The results of expert technical evaluation further showed that E1 and E2 had better technical movements than C1; were higher than C1 in the overall level of long jump skill learning, technical standardization, and skill evaluation; and had a higher proportion in high sections than C1. Moreover, the technical movements of E1 and E2 are more accurate, standardized, coordinated, and effective. Through further observation of the process record, it is found that C1 has always been in a “wavy” progress and high uncertainty in the overall development, while E1 and E2 are in a steady upward trend and in an “adjusting state” of steady growth. In the mode of health data-driven physical education, students can test and practice in a planned and targeted way in each lesson, thus achieving higher learning quality and significantly improving the acquisition of sports knowledge and the strengthening of exercise skills. Although the experiment period is not long, from the perspective of quality development, health data-driven physical education can relatively shorten the process of finding “problem state,” accelerate the learning process, further strengthen the combination of inside and outside class, improve the learning efficiency, and ultimately benefit the improvement of students' ability.

## 4. Development of Health Data-Driven Physical Education

### 4.1. Reshaping the Structural Relations of Physical Education Classroom Teaching Comprehensively by Quantitative Means

Quantitative means provide an analytical perspective and action basis for health data-driven physical education teaching. At present, the tracking and analysis technology of health data has been preliminarily applied in indoor physical education teaching by means of network or intelligent teaching system platform [31, 32]. This analytical technique generally includes three levels: technology, method, and application. On the technical level, the wearable devices and noncontact sensor technology can obtain real-time and non-real-time data on students' learning state, physical and mental performance, etc. Offline and online mathematical modeling technology can discover the fine construction process of discrete and nonlinear exercise and health knowledge of students in ability development stage and finally depict the development process of exercise with intuitive data visualization technology. On the method level, hybrid research methods combining dynamic process progress with static result state can deeply understand complex phenomena in exercise learning, perspective causes of exercise knowledge and skills, socioeconomic methods of macroscopic overall physical health and micro individual skill development, etc.; diagnose problems restricting the development of exercise ability according to learning style, behavior preference, and other factors; and then plan a learning path that meets the needs of the students. On the application level, the characteristics of physical education are reexamined from different subject perspectives according to the objectivity of health data, the laws of physical education are retraced from different time dimensions according to the continuity of health data, and the influence of physical education is reevaluated from different observation scales according to the scale of health data. Ultimately, the health data-driven physical education teaching with quantitative means provides teachers with comprehensive and whole-process teaching services and supports students to learn accurately, individually, and systematically.

With the important goal of improving physical education, effective and interactive exercise teaching mode is restricted by individual differences, diversity of exercise, instantaneity of exercise behavior, and subjectivity and objectivity of teaching. Teacher's control of teaching stays in a certain section and can only focus on students' limited physical behaviors. Most of the teaching process is dominated by visual observation, verbal communication, and skill evaluation, which easily leads to inadequate feedback and lack of communication [33]. The data cognition realized by data tracking redefines the teaching process with the help of abundant health data information. The flexible reorganization of the teaching process becomes reasonable and dependable, presenting the characteristics of dynamic process, in-depth monitoring, and intelligent regulation. Teaching is no longer limited to the preset static teaching design but can be carried out dynamically according to different people, circumstances, and materials. The objectives of physical education and the all-round development of students' personality are better realized, and a new form of effective physical education is established. Therefore, health data-driven physical education relies on a comprehensive and integrated teaching analysis process to strengthen the communication between teachers and students and restructure a new type of teacher-student relationship and classroom form.

### 4.2. Innovation of Decision-Making Model to Improve the Effectiveness and Quality of Physical Education Teaching Objectives

The decision-making mode determines the operational logic and objective thinking of health data-driven physical education. As a new teaching mode in the information age, the current health data-driven physical education teaching emphasizes problem-oriented more. With the objective presentation of health data, it causes students to think about the teaching situation; encourages students to learn and master systematized, structured, and standardized exercise knowledge and skills; and conforms to the cultivation concept of core quality of exercise discipline. Teachers should adhere to the concept of student-centered and technology-supported learning to provide students with more modern learning experience, improve students' information literacy, broaden students' vision of exercise and health, and improve the scientific and effective teaching. In the process of changing from experience-driven to health data-driven education, teachers need to have high data literacy, mainly reflected in the application of data to improve the knowledge base, thinking habits, and action ability of teaching [34]. However, teaching and learning are two-way interactive processes, and both teachers and students are interdependent and grow together. Under the guidance of health data perspective, the community of teachers and students focuses on specific exercise practice problems. Through scientific data mining, analysis, communication, and evaluation, it jointly explores reasonable and effective teaching decisions to deal with various problems, realizes simultaneous development, and finally achieves the goal of educating people by virtue.

With the deep integration of health data-driven learning and physical education, the existing teaching status will undergo subversive changes, and health data will gradually become the core label of new physical education. Exercise teaching needs to break the traditional ideas, and every member of the community of teachers and students needs to study and develop the corresponding data quality, including health data acquisition and data analysis. Health data-driven physical education not only realizes the orderly transformation of “health data-information-knowledge-skill,” but also realizes the communication and cooperation between members based on common language. Therefore, health data-driven physical education needs to rely on the two-way teaching interaction between teachers and students, so that the goals between teachers and students are more consistent; at the same time, the communication is more smooth, the community of teachers and students in physical education is more closely integrated, and the cultivation goal of core literacy of physical education is more effective and of high quality.

### 4.3. Health Data Feedback Promotes the Innovation and Development of Physical Education Concept

The feedback of health data reflects the core idea and future trend of health data-driven physical education. The key to achieving this requirement lies in the normal application of education and teaching and comprehensive innovation. A large number of experiences also show that physical education teaching needs to strengthen the combination with modern information technology, multimedia technology, and other fields to encourage students to form necessary exercise information literacy, sharp exercise information collection literacy, modern information technology communication ability, and necessary scientific and technological literacy in exercise learning [35]. Through the comparison of health data feedback, the students can individually and adaptively locate the best learning partners, thus optimizing the communication space among the community of teachers and students and accelerating the construction of students' equal exercise knowledge and ability. The continuous and consistent positive feedback of health data can help students form active exercise learning attitude, acquire basic knowledge and skills of exercise disciplines, and at the same time form correct exercise values, which also become the driving force for integration and innovation of physical education.

Superficially, health data-driven physical education continues to maintain the basic process structure of the course, but the support services achieved by health data feedback have been embedded in various physical education links. During the process of health data feedback, the advantages of health data in classroom teaching can be brought into play through data integration of various means, so that periodic accurate feedback exists in the whole process of learning, which changes the black-box learning mode of preschool test and post-school evaluation. Students can self-evaluate and improve, as well as understanding themselves from health data to optimize their learning strategies, methods, and abilities. Therefore, health data-driven physical education relies on periodic and whole-process health data feedback and carries out physical education reform from teaching mode, learning evaluation, educational decision-making, and learning quality, bringing opportunities and new life for physical education reform.

## 5. Conclusion

This paper studies health data-driven learning to promote the innovation and development of physical education teaching; constructs a health data-driven physical education teaching model; strengthens the collection, analysis, feedback, and utilization of data; and explains the specific ways of learning support design in each link based on health data in order to realize the deep integration of health data and physical education. Empirical study shows that health data-driven physical education teaching has a good effect on improving students' emotional attitudes and values, learning process and methods, knowledge and skills, etc. Furthermore, it is also helpful in the health management of the public environment. In the future exploration and development, the application of health data-driven learning-oriented innovation in physical education needs theoretical and practical two-way driven and comprehensive interpretation. It still needs to be tried in concept, method, technology, and means to provide rich theoretical guidance and practical reference for optimizing physical education teaching mode, providing strong support for comprehensively deepening the reform and innovation of physical education, and realizing the modernization of physical education.

## Figures and Tables

**Figure 1:** Framework of health data-driven physical education scheme.

**Table 1:** Performance of E1, E2, and C1 in health data-driven physical education.

Whether wearable devices affect learning	Average training time (one week)/h	Grade improvement (%)	Times of training	Confidence level (1–5)
No	1.56	38.06	1	4.61
Slightly	2.47	21.59	2	3.16
—	3.07	—	>3	2.09

## Data Availability

All data used to support the findings of the study are included within this paper.
